The article "miR-5089-5p suppresses castration-resistant prostate cancer resistance to enzalutamide and metastasis via miR-5089-5p/SPINK1/ MAPK/MMP9 signaling" was retracted in 2020. Reasons: unreliable results or conclusions; concerns about the results or conclusions.

# miR-5089-5p suppresses castration-resistant prostate cancer resistance to enzalutamide and metastasis via miR-5089-5p/SPINK1/ MAPK/MMP9 signaling

**DOI:** 10.18632/aging.103485

**Published:** 2020-07-21

**Authors:** Zhi-Chao Wang, Yan Li, Ke-Liang Wang, Lu Wang, Bo-Sen You, Dan-Feng Zhao, Zhong-Qing Liu, Rui-Zhe Fang, Jia-Qi Wang, Wei Zhang, Jin-Ming Zhang, Wan-Hai Xu

**Affiliations:** 1 Heilongjiang Key Laboratory of Scientific Research in Urology, The Fourth Affiliated Hospital of Harbin Medical University, Harbin 150001, China; 2 Department of Anesthesia, The Fourth Affiliated Hospital of Harbin Medical University, Harbin 150001, China

**Keywords:** castration resistant prostate cancer, miR-5089-5p, SPINK1, enzalutamide resistance, metastasis

## Abstract

Whether serine protease inhibitor Kazal type 1 (SPINK1) being associated with enzalutamide (Enz) resistance and metastasis of castration-resistant prostate cancer (CRPC) has not been clear. SPINK1 promoted Enz resistance by upregulating Androgen receptor splicing variant 7 (ARv7), and enhanced the invasion/migration of Enz-resistant cells via ERK/p38/ MMP9 signaling. Furthermore, miR-5089-5p suppressed SPINK1 mRNA through direct binding to its 3'UTR, and reversed its pro-proliferative and pro-metastatic effects. Mice bearing SPINK1-knockdown Enz-resistant PCa tumors showed significantly longer survival compared with those bearing wild-type tumors, while treatment with miR-5089-5p inhibitor abrogated the protective effects of SPINK1 knockdown. Taken together, SPINK1 can be used as a biomarker of resistance to Enz, and the miR-5089-5p/SPINK1/MAPK/MMP9 axis is a suitable therapeutic target against Enz-resistant and metastatic CRPC.

Methods: The expression of SPINK1 in Enz-resistant prostate cancer (PCa) cell lines was detected through next-generation sequencing data and metastatic PCa patients. In vivo and in vitro experiments were performed to investigate the role of SPINK1 in Enz-resistance and metastasis.

## INTRODUCTION

Castration-resistant prostate cancer (CRPC) is a stage of advanced prostate cancer and is associated with poor prognosis. American Food and Drug Administration recently approved an androgen receptor (AR)-targeting drug Enzalutamide (Enz, also known as MDV3100), which showed a significant inhibitory effect on CRPC cells and prolonged median overall survival by 4.8 months [1, 2]. Despite its survival benefits, not every patient responds to Enz and the responsive patients eventually develop resistance [3, 4]. In addition, its adverse effect is also associated with increased risk of neuroendocrine differentiation and metastasis. With widespread use, resistance to enzalutamide is a major clinical problem. Therefore, it is essential to identify the genes involved in Enz resistance through genome-wide profiling.

Serine protease inhibitor Kazal type 1 (SPINK1) is expressed in a variety of tissues and cells, which plays a variety of biological functions. Under physiological conditions, SPINK1 is mainly secreted by pancreatic acinar cells and inhibits abnormal activation of trypsinogen in pancreatic acinar and pancreatic duct. Under stress conditions such as severe blood loss, trauma and sepsis, SPINK1 is produced by the liver and released into the blood as an acute response protein. More importantly, SPINK1 can play an indispensable role as a growth factor in tissue differentiation and development in multiple cancers [5]. The serum concentration of SPINK1 in ovarian cancer patients is significantly increased, which can be used as a diagnostic indicator and can indicate the prognosis [6]. Hass HG et al. found that the mRNA level of SPINK1 in liver cancer cells significantly increased [7]. In addition, antagonists of androgen lead to elevation of SPINK1, which promoted EMT, stemness and cellular plasticity in prostate cancer [8]. However, the specific mechanism of SPINK1 has not been clear.

We identified SPINK1 as a key player in Enz resistance, which acts via upregulating ARv7. In addition, SPINK1 enhances the metastatic ability of PCa cells by activating ERK/p38/MMP9 signaling. We also identified miR-5089-5p as the transcription regulator of SPINK1, which abrogated the effects of the latter.

## RESULTS

### SPINK1 overexpression in PCa cells positively correlates with Enz resistance and metastasis

High-throughput sequencing showed consistently higher SPINK1 expression levels in the Enz-resistant cells (Figure 1A), which was verified in the C4-2R and C4-2B-R cells by qRT-PCR and Western blotting (Figure 1B, 1C). Consistent with the literature reports on SPINK1 overexpression in metastatic PCa patients [9], high levels were also confirmed in our 24 clinical samples (Figure 1D), and significantly associated with overall survival (*P*=0.0039; data from our hospital) (Figure 1E). Analysis of the GEO dataset GDS2545 showed higher SPINK1 expression in metastatic PCa tissues compared to primary PCa and normal prostate tissues (Figure 1F). Kaplan-Meier analysis of the TCGA dataset (http://cancergenome.nih.gov/) further showed that SPINK1 overexpression was significantly associated with decreased overall survival (Figure 1G). Taken together, SPINK1 acts as an oncogene in PCa, and promotes Enz resistance and metastasis.

**Figure 1:** **SPINK1 expression levels in Enz-resistant cells and metastatic PCa patients.** (**A**) Differentially expressed genes (DEGs) between Enz-sensitive cell and Enz-resistant cell lines (≥ 5-fold and *P*< 0.001). The columns represent individual genes and rows indicate the cell lines. Red and blue color represent high and low expression respectively (**B**) Western blot showing high SPINK1 protein levels in C4-2R and C4-2B-R (**C**) RT-PCR results showing high SPINK1 mRNA levels in C4-2R and C4-2B-R. (**D**) Representative IHC images showing *in situ* SPINK1 expression in human PCa tissues. Positive SPINK1 expression was significantly associated with worse overall survival (*p*=0.0039, log-rank test, data from our hospital). (**E**) GDS2545 dataset results showing SPINK1 mRNA levels in the normal prostate tissues, and primary and metastatic prostate tumors. (**F**, **G**) Kaplan-Meier plot showing survival rate of SPINK1^hi^ and SPINK1^lo^ PCa patients in the TCGA dataset, SPINK1^hi^ is associated with poor prognosis (*p*=0.0018).

### SPINK1 increases Enz resistance by upregulating the androgen receptor splicing variant 7 (ARv7)

To determine the mechanism underlying SPINK1 action in Enz-resistant PCa, we generated stable SPINK1-knockdown (shSPINK1) C4-2R and C4-2B-R cells, and SPINK1-overexpressing (oeSPINK1) C4-2 and C4-2B cells (Figure 2A). The C4-2R and C4-2B-R cells were indeed resistant to Enz, as indicated their high proliferative rates in the presence of the drug, which was significantly inhibited upon SPINK1 knockdown (Figure 2B, 2C). Consistent with a previous study implicating ARv7 in Enz resistance [4], we demonstrated a direct interaction between SPINK1 and ARv7 through co-IP (Figure 2D). Furthermore, SPINK1 overexpression in the Enz-sensitive cells increased ARv7 levels, whereas Enz-resistant cells showed a downregulation in ARv7 following SPINK1 knockdown (Figure 2E, 2F). Taken together, SPINK1 likely promotes Enz-resistance via ARv7.

**Figure 2:** **SPINK1 promotes Enz resistance and production of ARv7.** (**A**) Western blots and RT-PCR results validating SPINK1 knockdown in C4-2R and C4-2B-R cells, overexpression in C4-2 and C4-2B cells. (**B**) Percentage of viable +/shSPINK1 C4-2R and C4-2B-R cells with/without Enz treatment. (**C**) Edu incorporation rate in +/shSPINK1 C4-2R and C4-2B-R cells with/without Enz treatment. (**D**) Immunoblot showing co-immunoprecipitation of SPINK1 and ARv7 in the C4-2R cells. (**E**, **F**) Western blots and qRT-PCR results showing AR-v7 protein and mRNA levels in oeSPINK1 C4-2 and C4-2B cells, and shSPINK1 C4-2R and C4-2B-R cells.

### SPINK1 promotes metastasis via the MAPK/MMP9 signaling pathway

The *in vitro* migration and invasiveness of the PCa cell lines were determined by wound healing and transwell assays respectively. While SPINK1 knockdown significantly inhibited the migration and invasion of the Enz-resistant cell lines, the C4-2 and C4-2B cells showed enhanced migrations and invasiveness following SPINK1 overexpression (Figure 3A–3D). However, TCGA data on PCa tissues did not show any correlation between SPINK1 expression levels and that of ki67 and MMP9, which are respectively associated with high tumor cell proliferation and metastasis. In contrast, the GEO dataset showed that SPINK1 overexpression was positively correlated with high levels of ki67 and MMP9 expression, especially in the metastatic PCa tissues (Figure 3E, 3F). To further explore the possible mechanisms underlying SPINK1-induced metastasis, we analyzed the ERK and p38 signaling pathway. The p-ERK and p-p38 levels were significantly inhibited in the shSPINK1 C4-2R and C4-2B-R cells (Figure 3G, 3H), and upregulated in the oeSPINK1 C4-2 and C4-2B cells (Figure 3I, 3J). Taken together, the pro-metastatic effects of SPINK1 are likely mediated via the ERK/p38 pathway.

**Figure 3:** **SPINK1 enhances migration and invasion of Enz-resistant cells via MAPK/MMP9 signaling.** (**A**, **B**) Migration rates of shSPINK1 C4-2R and C4-2B-R cells, and oeSPINK1 C4-2 andC4-2B cells in the wound healing assay. (**C**, **D**) Invasive capacity of shSPINK1 C4-2R and C4-2B-R cells, and oeSPINK1 C4-2 and C4-2B cells in the transwell assay. (**E**, **F**) Correlation of SPINK1 expression with MMP9 and Ki67 levels in PCa tissues of TCGA and GSE66187 datasets. (**G**–**J**) Relative p-ERK, p-p38, Ki67 and MMP9 protein levels in shSPINK1 C4-2R and C4-2B-R cells, and oeSPINK1 C4-2 and C4-2B cells. Each bar represents the mean ± SEM, *P < 0.05; **P < 0.01; ***P < 0.001.

### MiR-5089-5p abrogates the pro-neoplastic effects of SPINK1 on PCa cells

To elucidate the mechanisms underlying SPINK1 upregulation in Enz-resistant PCa cells, we predicted potential targeting miRNAs using the Target Scan and miRmap algorithms, and identified miR-5089-5p, miR-892c-5p and miR-4694-3p as putative candidates (Figure 4A). Further validation in the C4-2R and C4-2B-R cells indicated that only miR-5089-5p was significantly down-regulated in the Enz-resistant lines (Figure 4B). Luciferase reporter assay further showed that the miR-5089-5p mimic controlled SPINK1 promoter activity (Figure 4C). In addition, miR-5089-5p inhibitor and mimic respectively increased and decreased SPINK1 mRNA expression levels (Figure 4D). To explore the role of the miR-5089-5p-SPINK1 axis on Enz-resistant PCa, we then analyzed the biological effects of manipulating the miRNA. While the miR-5089-5p mimic partially blocked SPINK1-mediated invasion and migration, miR-5089-5p inhibitor partially reversed the block on cell invasion and migration in shSPINK1 C4-2R cells (Figure 4E–4H). Finally, inhibition of miR-5089-5p also restored ARv7 levels in the shSPINK1 C4-2R cells (Figure 4I, 4J).

**Figure 4:** **SPINK1 enhances Enz resistance and metastasis via miR-5089-5p inhibition.** (**A**) Venn diagram (left panel) of SPINK1-targeting miRNAs predicted by miRmap and Targetscan. Putative miR-5089-5p binding sites on the 3′-UTR of SPINK1 (right panel). (**B**) qRT-PCR results showing differential expression of miR-5089-5p in C4-2R/C4-2B-R compared to C4-2/C4-2B cells. (**C**) Luciferase reporter construct with the wild-type or mutated SPINK1 3’UTR downstream of the firefly luciferase reporter gene (left panel). Luciferase reporter activity in HEK293T cells co-transfected with the respective constructs along with miR-5089-5p mimics (right panel). (**D**) SPINK1 mRNA levels in cells treated with the miR-5089-5p inhibitor and miR-5089-5p mimic. (**E**, **F**) The migration abilities of +/ shSPINK1 and +/ miR325p inhibitor C4-2R cells (upper panels), and +/ oeSPINK1 and +/ miR-5089-5p mimic C4-2 cells (lower panels) in the wound healing assay. Percentage of migrating cells are on the right panels. (**G**, **H**) The invasiveness of +/ shSPINK1 and +/ miR325p inhibitor C4-2R cells (upper panels), and +/ oeSPINK1 and +/ miR-5089-5p mimic C4-2 cells (lower panels) in transwell assay. Percentage of invading cells are on the right panels. (**I**) ARv7 protein levels in +/oeSPINK1 and +/miR-5089-5p mimic C4-2 cells (upper panels), and +/ shSPINK1 and +/ miR325p inhibitor C4-2R cells (lower panels). Relative protein levels are shown on the right. (**J**) ARv7 mRNA levels in +/oeSPINK1 and +/miR-5089-5p mimic C4-2 cells (upper panels), and +/ shSPINK1 and +/ miR325p inhibitor C4-2R cells (lower panels).

### The miR-5089-5p-SPINK1 axis modulates the growth of Enz-resistant PCa tumors in vivo

To confirm the *in vitro* findings, we established a subcutaneous PCa model in mice using +/shSPINK1 C4-2R cells. After inoculation, the shPINK1-C4-2R tumor-bearing mice showed prolonged survival compared to the mice with wild-type C4-2R tumors. However, treatment with miR-5089-5p inhibitor reversed the protective effects of SPINK1 knockdown, thereby promoting Enz-resistant tumor growth and decreasing survival duration (Figure 5A–5D). Furthermore, the tissues of shSPINK1-C4-2R tumors show low *in situ* expression of SPINK1, MMP9 and ki67, which was rescued by miR-5089-5p inhibition (Figure 5E).

**Figure 5:** **Role of miR-5089-5p and SPINK1 in Enz resistance and metastasis in vivo.** (**A**) Representative images of tumor xenografts excised from mice implanted with Enz-resistant cells with/without miR-5089-5p inhibitor treatment. (**B**, **C**) Tumor volumes and weight of different groups. (**D**) Survival rate of tumor-bearing mice of different groups (*p*=0.05, Kaplan-Meier). (**E**) In situ expression levels of SPINK1, ki67 and MMP9 in the tumor tissues (Scale bar—100 μm; The top right corner, Scale bar—50 μm).

## DISCUSSION

Enz as the second-generation antiandrogen has significantly improved the clinical outcome of CRPC patients. However, a significant proportion of the patients eventually develop drug resistance and/or metastasis after long-term Enz treatment, likely due to presence of both AR+ and AR- cells in the tumors, and the possible activation of AR–dependent or independent pathways resulting in cancer progression [10–22]. Several mechanisms of CRPC resistance to androgen deprivation therapy (ADT) have been proposed, including constitutive activation of ARv7 [10], ARF876L mutation [14, 15], AR amplification and overexpression [16], altered steroidogenesis [17], upregulation of the glucocorticoid receptor [18], and AKT signaling [22], of which ARv7 induction is supported by the strongest clinical data. The clinical study revealed that CRPC patients with detectable ARv7 in circulating tumor cells had poor responses to ADT-Enz [4]. Furthermore, ARv7 might be linked to bone metastases in CRPC [23]. These clinical data point to the possible reason why ADT-Enz may always fail due to ARv7 induction. In our study, high throughput sequencing of Enz-sensitive and the parent Enz-resistant cell lines revealed 3945 resistance-related genes, including SPINK1 which is often overexpressed in Enz-resistant PCa cell lines. Furthermore, we found that SPINK1 directly bound to and upregulated ARv7, and mediated Enz resistance.

SPINK1 is normally expressed in the liver, pancreas, colon, and other gastrointestinal organs, while aberrantly high expression levels have been reported in cancers of the prostate, lung, bladder, pancreas, colon, ovaries, gastric organs, liver and breast [6, 7, 24–30]. SPINK1 overexpression is associated with poor prognosis in general, and specifically with the Gleason grade, proliferation, and neuroendocrine differentiation in primary prostate cancers [31, 32]. In addition, its expression levels increase further with the progression from primary tumors to CRPC [33], and correlate with aggressiveness and recurrence [27, 30, 34–36]. At present, SPINK1 may represent a molecular subtype of prostate cancer [37]. However, it is not clear whether SPINK1 promotes PCa metastasis, especially in patients treated with ADT-Enz. In our study, SPINK1 is overexpressed in metastatic prostate cancer patients and associated with poor survival, and knocking down SPINK1 in the Enz-resistant cells significantly decreased their migration and invasiveness, and opposite effects were seen following SPINK1 overexpression in the Enz-sensitive cells. Another major finding of our study was SPINK1-mediated upregulation of MMP9, one of the matrix metalloproteases (MMPs) that degrade the extracellular matrix and promote tumor cell invasion and metastasis through the MAPK signaling pathway [38, 39]. High expression of MMPs, especially MMP-9, is associated with increased metastatic potential in several human cancers, including prostate cancer [40–44]. Two previous studies have indicated the involvement of MMP9 in the higher metastasis and invasiveness of PCa [45, 46]. Therefore, we hypothesized that MMP9 also plays a crucial role in promoting metastasis in Enz- resistant PCa cells. Mechanism dissection revealed that SPINK1 mediate pro-metastatic effects in the Enz-resistant cells via ERK/p38/MMP9 signaling.

Several studies have shown that members of the miR-200 family, including miR-452-5p and miR-34a, are significantly involved in chemo-resistance [47–49]. Besides, miRNAs are promising therapeutic target for clinical application. We identified miR-5089-5p as a key post-transcriptional regulator of SPINK1, which not only downregulated SPINK1 but also inhibited the migration and invasion of the Enz-resistant PCa cells. Therefore, the miR-5089-5p-SPINK1 regulatory axis is a novel therapeutic target against Enz-resistant and metastatic PCa.

In summary, SPINK1 promotes Enz resistance by upregulating ARv7 and enhances the metastatic ability of the Enz-resistant cells through ERK/p38/MMP9 activation. SPINK1 can be used as a biomarker in Enz-resistant PCa. The miR-5089-5p-SPINK1 regulatory axis also is a potential therapeutic target in Enz-resistant PCa. (Figure 6)

**Figure 6:** **The miR-5089-5p-SPINK1 mediates Enz resistance by upregulating ARv7 and the miR-5089-5p-SPINK1/MAPK/MMP9 axis mediates metastasis.** Enz treatment increase the expression of SPINK1 in Enz-resistant prostate cancer cells, which was negatively regulated by mirna5089-5p. Aberrantly high levels of SPINK enhances Enz resistance by upregulating ARv7, and promotes migration and invasion via ERK/p38/MMP9 signaling.

## MATERIALS AND METHODS

### Patients and samples

Prostate cancer (PCa) tissue specimens were collected from patients with definite histo-pathological diagnosis who underwent prostate biopsy or prostatectomy at the Forth Affiliated Hospital of Harbin Medical University. All samples were further confirmed by two pathologists blinded to patient data. The study was approved by the Institutional Review Board, and informed consent was obtained from all patients.

### Reagents

Anti-actin (10366-1-AP) was purchased from Proteintech (USA), anti-ki67 (WL01384a) antibody from Wanleibio Technology (China), anti-SPINK1 (sc-374409) and anti-MMP9 (sc-21733) antibodies from Santa Cruz Biotechnology (USA), and anti-p-ERK (Thr202/Tyr204), anti-ERK (137F5), anti-p-p38 (Thr180/Tyr182), anti-p38 (D13E1) and anti-ARv7 (E3O8L) antibodies from Cell Signaling Biotechnology (USA). The miR-5089-5p inhibitor and miR-5089-5p mimic were bought from GenePharma (China). The pLKO.1-shSPINK1 and pWPI-oeSPINK1 plasmids were synthesized and packaged according to the protocol.

### Cell culture

The human PCa cell lines C4-2 and C4-2B cells (from ATCC) were cultured with Enz for 3 months, starting with 10μM and steadily increased by 10μM every 20 days to 40μM. The ensuing Enz-resistant cells – designated C4-2R and C4-2B-R respectively – were maintained in RPMI 1640 (BI) medium with 10μM and 20μM Enz.

### MTT assay

The cells were seeded in 24-well plates at the density of 5000 cells/well/600μl media, and treated with DMSO or 10mM Enz for 0, 1, 2 and 4 days. To determine cell viability at each time point, 300μl of the MTT reagent (Sigma, Germany) was added to each well, and the cells were incubated for 2h. The medium was then removed, and 300μl DMSO was added to dissolve the formazan crystals. The optical density at 490 nm was measured by a microplate reader (BioTek, USA).

### EDU assay

The SPINK1-knockdown and control cells were seeded into six-well plates, and treated with DMSO or 10mM Enz for 24h. EdU and Hoechst staining was performed as per the instructions of an EdU-labeling kit (RiboBio, Guangzhou, China). The EdU-positive cells were counted in five random fields under a fluorescence microscope.

### Cell invasion assay

The *in vitro* invasiveness of the Enz-resistant PCa cells was determined by the transwell assay. The suitably-treated cells were harvested and seeded at 5×10^4^ cells/well with serum-free media into the Matrigel (BD Corning, USA)-coated upper transwell chambers, and the lower chambers were filled with 750μl complete medium. After a 24h incubation, the invading cells present on the lower surface of the membranes were fixed by 4% paraformaldehyde and stained with 0.1% (w/v) crystal violet. The number of invaded cells were counted in ten randomly chosen fields at 100x magnification, and the assay was repeated thrice.

### Wound healing assay

The migration capability of the cells was determined by the wound healing assay. Briefly, the cells were seeded into 6-well plates and cultured till 70%~80% confluency. The monolayers were scratched with sterile 200μl pipette tips, and rinsed with PBS. The “wound” area was imaged at 0, 24 and 48h post-scratching, and the number of migrating cells were counted.

### RNA extraction and qRT-PCR

Total RNA was extracted using Trizol reagent (Invitrogen, USA), and 1μg per sample was reverse transcribed using ReverTra Ace qPCR RT Kit (TOYOBO, Japan). Quantitative RT-PCR was conducted using Applied Biosystems 7500 Fast Real-Time PCR System with SYBR green (TOYOBO, Japan), and the expression levels of the genes of interest were normalized to that of GAPDH and U6.

### Western blotting

Cells were lysed in RIPA buffer, and 20-40μg protein per sample were separated by 8–10% SDS-PAGE, and transferred onto NT membranes (PALL, Gelman Laboratory). After blocking, the membranes were sequentially incubated with primary and HRP-conjugated secondary antibodies, and protein bands were visualized using the ECL system (Wanleibio, China).

### Luciferase assay

The cells were seeded into 12-well culture plate at 50% confluency. After culturing for 16h, the cells were transfected with cDNA, miR-5089-5p mimic, or miR-NC using Lipofectamine 2000 (Invitrogen). Luciferase activity was measured using Dual-Luciferase Assay (Promega, Madison, WI, USA) 48h after transfection as per the manufacturer’s instructions. Three replicates were tested per sample, and pRL-TK was used as the internal control.

### Co-Immunoprecipitation (CO-IP) assay

The suitably-treated cells were harvested and washed twice with cold PBS, and lysed in cold RIPA buffer. After centrifuging the lysates, the supernatant was aspirated and incubated overnight at 4°C with 2 mg anti-IgG, anti-SPINK1 or anti-ARv7 antibodies. After adding 100μl Protein-A/G–agarose beads (Santa Cruz Biotechnology, USA), the reaction mixes were shaken overnight at 4°C. The immune complexes were then precipitated, washed thrice with PBS, and boiled for 5 mins with 2x SDS-PAGE loading buffer. The immuno-precipitates were resolved by 10% SDS-PAGE, followed by Western blotting with antibodies against SPINK1 and ARv7.

### Immunohistochemistry (IHC)

Tissue specimens were fixed, embedded in paraffin, and cut into 5μm sections. The latter were first treated with EDTA for antigen retrieval, and then with 3% hydrogen peroxide to quench endogenous HRP activity. To block non-specific binding, the sections were blocked in goat serum for 10 minutes at room temperature, followed by overnight incubation with primary antibodies against SPINK1 (1:50, Santa Cruz, sc-374409), MMP9 (1:50, Santa Cruz, sc-21736) and ki67 (1:100, Wanleibio, WL01384a, Shen Yang, China) at 4°C. A rabbit two-step assay kit (PV-6001, ZSGB-BIO, Bei Jing, China) and DAB (ZLI-9018, ZSGB-BIO, Bei Jing, China) were respectively used to label and detect HRP, and the sections were counter-stained with Mayer’s hematoxylin.

### In *vivo* tumorigenesis assay

Eighteen male athymic BALB/c nude mice (Beijing Vital River Laboratory Animal Technology Co. Ltd., China) were randomly divided into three groups: C4-2R, shSPINK1 C4-2R and shSPINK1 C4-2R + miR-5089-5p inhibitor. The respective cells (4 x10^6^) were mixed with Matrigel (1:1) and injected subcutaneously into the flanks, and once the tumor grew to 50 mm^3^, 10nM of the miRNA inhibitor (in 0.1 ml saline) was locally injected into the designated mice once every 3 days for 2 weeks. The tumors were measured using calipers twice a week, and tumor volumes were calculated as length * width^2^/2. After four weeks, the tumors were harvested for further assays. All animal experiments were performed in accordance with the approved guidelines, and were approved by the institute.

### Statistical analysis

All statistical analyses were conducted using GraphPad Prism. Different groups were compared by ANOVA or Student’s t test as appropriate. The survival rates were estimated using the Kaplan-Meier method, and compared using the log-rank test. All experiments were repeated at least thrice, with each condition in triplicates. P values of *P < 0.05; **P < 0.01; ***or ****P < 0.001 were considered statistically significant.

### Availability of data and materials

The data generated or analyzed during this study are included in this article, or if absent are available from the corresponding author upon reasonable request.

## Supplementary Material

Supplementary Figures
